The article "Research on Fuzzy Comprehensive Evaluation Index System of Mental Health Education for College Students" was published in 2022. Journal: J Healthc Eng.

# Research on Fuzzy Comprehensive Evaluation Index System of Mental Health Education for College Students

**DOI:** 10.1155/2022/7106926

**Published:** 2022-04-18

**Authors:** Tao Wang

**Affiliations:** Eastern Liaoning University, Dandon, Liaoning 118000, China

## Abstract

With the economic development and social progress, psychological crisis has become a very serious social problem, and the university campus is also inevitably affected. College students' ability to resist pressure is poor, their psychology fluctuates greatly and changes constantly, and they are easily influenced by the outside world. Mental health assessment is a scientific means to quantitatively analyze and infer the characteristics of psychological changes in people's behaviors by measuring and observing people's representative behaviors in a strictly controlled environment. Analytic hierarchy process (AHP) is a method to determine the relative importance weight and relative order of advantages and disadvantages of various factors in the system, while fuzzy comprehensive evaluation is an effective method to evaluate fuzzy things comprehensively. This paper introduces the principle of the fuzzy comprehensive evaluation method, analyzes the feasibility and applicability of the fuzzy comprehensive evaluation method in social work evaluation of college students' mental health schools, and draws relevant research conclusions and suggestions.

## 1. Introduction

With rapid social change, rapid economic growth, increasingly fierce competition and the diversification of cultural values, the growth of college students is under pressure from all aspects, and their psychological problems are complicated and changeable [1]. In recent years, with economic development and social progress, psychological crisis has become a very serious social problem; the university campus is also inevitably affected [2]. College students are facing increasing pressure from competition, the economy, study, employment, and emotions, and they are more likely to encounter or produce various psychological problems [3]. Today's world is in an era of fierce competition. The essence of competition is the competition of high-quality human resources. College students are the reserves of national development. They want to survive, develop, and succeed in this increasingly competitive society, so education shoulders the responsibility of cultivating high-quality talents [4]. At this stage of life, special groups of college students are in the most important and critical stage of life. At this stage, they are full of passion and vitality. However, they have a poor ability to resist pressure, and their psychological fluctuation is large and constantly changing. They are easily affected by the outside world. If they do not solve their psychological problems in time, it will have an impact on their lives and studies and cannot integrate into society [5].

Mental health school social work is actually a combination of traditional school mental health education and school social work. Mental health education is very important for the healthy growth of college students [6]. The establishment and development of college students' mental health evaluation system and targeted psychological counseling for college students to master their psychological development track is the top priority of college mental health education [7]. In order to correct the status of mental health education in the overall education, schools must strengthen and improve mental health education so that students can learn and live well in school, and at the same time, their physical and mental health and other specialties can be fully developed and cultivated [8]. Therefore, it is easier to evaluate the mental health of college students [9]. Analytic hierarchy process (AHP) is a method to determine the relative importance weight and relative priority order of each factor in the system, and fuzzy comprehensive evaluation is an effective method for multifactor comprehensive evaluation of fuzzy things [10].

This paper is divided into four parts. The first part expounds the research background and relevant literature references. The second part expounds the fuzziness of the performance evaluation of mental health education in colleges and universities and the uncertainty of the evaluation scope. The third part expounds the fuzzy comprehensive evaluation index system of mental health education. Finally, the full text is summarized.

## 2. The Fuzziness of Performance Evaluation Content and the Uncertainty of Evaluation Scope of Mental Health Education in Colleges and Universities

The fuzziness of the content and the uncertainty of the evaluation scope of the performance evaluation of mental health education in colleges and universities make it very difficult to objectively evaluate it. The psychological quality of contemporary college students not only affects their own development but also affects the normal operation of schools, which is also related to the improvement of the quality of the whole person. Psychological consultation plays a great role in treating their mental health and optimizing students' psychological quality, but it also has some limitations. According to the different personality characteristics of each individual student, we can accurately analyze and grasp the psychological changes of college students in environmental management colleges in China at different levels and stages, provide psychological health counseling for college students, and show interactivity in the counseling process. In the evaluation of the effects of mental health education in colleges and universities, the explicit, direct, and short-term effects are easy to notice and evaluate. The recessive, indirect, and long-term effects are often ignored by people, and it is difficult to evaluate them in practice [11]. School social work is to apply the theories, principles, and methods of social work improve the school learning environment and conditions, help students with difficulties to improve their ability to adapt to study and life, and overcome the difficulties in their growth to achieve the goals of personal socialization and school education.

The professional concept of school social work is people-oriented, helping others and helping themselves, and its aim is service. To publicize the knowledge of mental health care and mental health among college students and to make them understand their own psychological situation through various means such as online answering questions, testing, and consultation, especially for students with mental disorders, so as to realize their self-management and self-repair ability through the mental health assessment system. Although the country has issued a series of laws and regulations, schools attach different importance to them and develop in different situations. Schools that do not pay attention to mental health education have little capital investment and some wrong cognitions, so they only stay in form but do not really implement it in order to cope with the inspection. The shaping of students' mental health is a systematic project, including classroom teaching, extracurricular activities, teaching management, logistics services, and even family and society, so it is impossible to attribute all their achievements to the work of mental health educators. Of course, the performance evaluation of mental health education in colleges and universities must include the improvement of students' psychological status, but it is a difficult problem to solve. The quality of the college students' mental health education team largely determines its effectiveness. Mental health education requires highly qualified professionals. However, China's overall mental health education is not highly specialized. In addition, the number and quality of mental health educators make it difficult to meet the needs of development due to the unstable team of psychological tutors in various schools.

For fuzzy and unclear problems determined by multiple factors or defined by standards, each factor is evaluated separately by using the grade index and weight of evaluation factors, and each factor is comprehensively described by using the principle of membership degree, and a discriminant model is established to obtain the grade result to which the evaluation object belongs. The design of the evaluation index system is the basis of the effectiveness of the fuzzy comprehensive evaluation method, and its basic approach is to decompose the target layer by layer to form an index system according to certain standards. The evaluation system of mental health education in colleges and universities refers to the overall structure of indicators which can reflect the effect of mental health education in colleges and universities. Although the mental health education workers are exhausted, the students do not appreciate these activities. They think that these activities are only forms, which cannot solve their confusion, and that mental health education is only for people with serious psychological problems. The performance evaluation of the main body of mental health education in colleges and universities includes the improvement of the mental health level of the educated, the psychological influence of the educated on others, the quality and structure of the educators, and the improvement of the mental health level of the educators themselves after the completion of a mental health education activity [12]. The performance evaluation of the implementation process of mental health education in colleges and universities mainly includes the systematicness of mental health education plans, the scientificity of procedures and the creativity of methods, the collection and management of mental health education information, and the analysis and application of mental health education information. The standard of mental health is not only an ideal one, but also a vague one. Everyone may have shortcomings in front of these standards. For different individuals, mental health is different, so mental health is relative.

## 3. Fuzzy Comprehensive Evaluation Index System of Mental Health Education

As friends of college students, counselors can intervene in college students' problems with an equal status. This unique role and position will play a better guiding and supporting role in solving college students' psychological problems. In order to make the evaluation of the mental health education system in colleges and universities effective, it should be carried out according to the following steps: first, analyze the system according to the goals and functions of the mental health education system in colleges and universities and determine the evaluation index system. Secondly, a single evaluation is performed to obtain the degree of realization of the system under the corresponding evaluation indexes, and the realization values of different dimensions under different indexes are normalized to obtain the fuzzy matrix.

Table 1 shows fuzzy numbers and their numerical characteristics. Let the fuzzy number *x* represent an interval here, and each fuzzy number *x* can be represented by 3 certain numbers (*a*1, *a*2, *a*3), and its membership function as follows:

(1) $$\begin{array}{c} \mu_{A}\left\{\begin{array}{c} 0\\ \frac{x-a}{a_{2}-a_{1}}\;x\langle \;a_{1}\\ a_{1}\leq x<a_{2}\\ a_{2}\leq x\leq a_{3}\\ \frac{a_{3}-x}{a_{3}-a_{2}}\;x\rangle \;a_{3} \end{array}\right\}. \end{array}$$

The steps of the fuzzy analytic hierarchy process are summarized as follows: (1) constructing an analytic hierarchy process model; (2) using fuzzy numbers 1, 3, 5, 7, and 9 to identify the element values in the judgment matrix; and (3) multiply the relative weight *W*_*i*_ of each criterion with each element in the judgment matrix *a*. A new matrix is obtained as follows:

(2) $$\begin{array}{c} A\left\{\begin{array}{c} W_{1}\cdot x_{10}\;W_{2}\cdot x_{11}\;\ldots \;W_{n}\cdot x_{n}\\ W_{1}\cdot x_{20}\;W_{2}\cdot x_{21}\;\ldots \;W_{n}\cdot x_{2n}\\ \ldots \;\ldots \;\ldots \\ W_{1}\cdot x_{n0}\;W_{2}\cdot x_{2n}\;\ldots \;W_{n}\cdot x_{nn}. \end{array}\right.. \end{array}$$

The information of students' learning activities is fed back to the personalized data analysis module, and then reprocessed by the personalized data analysis module to update the student information base. Calculating information gain is the most common method. In the formula for calculating information gain, the information gain degree is as follows:

(3) $$\begin{array}{c} P=P\left(Y=1\right)\\ =F\left(\beta_{i}X_{i}\right). \end{array}$$

According to the idea of a decision tree, relevant data are obtained to describe in detail the method of obtaining information gain:

(4) $$\begin{array}{c} R_{t}\left(p_{1t},Q_{t}\right)=p_{1t}\cdot \min\left(I_{t}+Q_{t},D_{t}\right)-\left(p_{0t}\cdot Q_{t}+C_{t}\cdot AI_{t}\right)+R_{t-1}. \end{array}$$

Thirdly, make a comprehensive evaluation. According to the index system, the comprehensive evaluation value of a single index, the comprehensive category index, and the total evaluation value of the system are calculated in turn. These two methods have good application value in college students' mental health education. School case social work refers to the professional method of social work for college students; that is, school social workers use professional knowledge and technology of people and society to coordinate various available social resources and provide one-to-one services for students, aiming at helping college students fully understand their own resources and potential, improving themselves, and enhancing their ability to solve difficulties so as to achieve good adaptation to society and environment [13].

As an implicit ability that can activate athletes' internal potential, psychological skill plays an important role in training and competition, as well as technical and tactical ability. With the expansion of the coping research field and continuous observation of the increasingly prominent role of coping in competitive sports, it is necessary for us to have a deeper understanding of the complex relationship between coping and sports performance.  Table 2 shows a variance analysis of coping strategies at different exercise levels.

An athlete's mental behavior operation model is often described by a first-order differential equation, which can simulate the law of multilayer perception network over time. The following functional expressions are generally used to express the nonlinear characteristics of the network:

(5) $$\begin{array}{c} p\left(x\right)=KBy\left(x\right)-GB\frac{{\text{d}}^{2}y\left(x\right)}{\text{d}x^{2}}. \end{array}$$

According to mathematical ideas, obtain relevant data to describe in detail the method of obtaining information gain:

(6) $$\begin{array}{c} E=\frac{t_{m}+t_{u}}{\left(t_{m}/E_{m}\right)+\left(t_{u}+E_{u}\right)}\rho . \end{array}$$

The mental health of college students is not only related to studies, but also related to all aspects of life. College students are at a turning point in their lives. Colleges and universities should strengthen their mental health education and ideological education, guide them to form a correct world outlook, outlook on life and values, and make them adapt to society. At present, the psychological problems of college students are complicated and changeable. Different individuals must be involved in one-to-one or many-to-one working modes. The application of this method makes the mental health education of college students highlight and has strong pertinence. College students' mental health assessment is the guidance and foundation of college students' mental health education, so colleges and universities should put college students' mental health assessment first, improve the subjects of college students' mental health assessment, and establish a set of more scientific assessment standards [14]. The intervention of school group work emphasizes people's utility in the situation. This method is discussed from the commonness of recipients. It is believed that the problems faced by recipients have similarity rivers to organize these similar groups and form groups or groups to concentrate on solving the problems faced by individual members through the strength of groups, the interaction of group members, the process of groups, or the assistance of group workers.

## 4. Conclusions

The mental health of college students is not only related to studies, but also related to all aspects of life. College students are at a turning point in their lives. Colleges and universities should strengthen their mental health education and ideological education, guide them to form a correct world outlook, outlook on life and values, and make them adapt to society. The correct evaluation of the performance of mental health education in colleges and universities is an essential part of the process of mental health education. It reflects the actual effect of the implementation of mental health education in colleges and universities, which not only lays a foundation for educators to sum up experiences and lessons and further implement mental health education in colleges and universities, but also provides an objective basis for properly evaluating the work achievements of mental health educators. College students' mental health assessments are the guidance and foundation of college students' mental health education. Therefore, colleges and universities should put college students' mental health assessment first, improve the subjects of college students' mental health assessment, and establish a set of more scientific assessment standards. The evaluation index system of mental health education based on fuzzy comprehensive evaluation not only reduces the workload of manual measurement, but also shortens the time and makes the measurement results more scientific, which provides a better platform for moral education. In the daily mental health education of college students, college teachers should be good at combing the psychological and ideological problems of college students, integrating them together, guiding and educating college students, and providing them with timely help. However, this paper does not compare with the actual survey data, which makes the evaluation of college students' mental health has some limitations. This needs to be further strengthened in the future.

## Figures and Tables

**Table 1:** Fuzzy numbers and their digital characteristics.

Fuzzy number	Digital features

1	(1, 1, 3)
*x*	(*x* − 3, *x*, *x* + 2) *x* = 3, 5, 7
9	(7, 9, 11)

**Table 2:** Analysis of variance of coping strategies for different exercise levels.

Sports grade	*F*	Sig.

Centralized solution	1.425	0.308
Avoidance coping	2.152	0.225
Beyond coping	2.337	0.192

## Data Availability

The data used to support the findings of this study are included within the article.
